RETRACTED

# Sappanone A Alleviated IL-1*β*-Induced Inflammation in OA Chondrocytes through Modulating the NF-*κ*B and Nrf2/HO-1 Pathways

**DOI:** 10.1155/2022/2380879

**Published:** 2022-09-16

**Authors:** Zhi Zhang, Nan-Zhi Zhang, Meng Li, Dang-Feng Zhang, Xing Ma, Shuang-Li Zhou, Yu-Sheng Qiu

**Affiliations:** Department of Orthopaedics, The First Affiliated Hospital, College of Medicine, Xi'an Jiaotong University, Xi'an, 710061 Shaanxi, China

## Abstract

**Objective:**

This study was to examine the anti-inflammatory effect of sappanone A on interleukin- (IL-) 1*β*-stimulated osteoarthritis (OA) chondrocytes.

**Methods:**

Chondrocytes were pretreated with sappanone A for 2 h before subsequent IL-1*β* stimulation. The mRNA expression levels of iNOs, COX-2, aggrecan, and collagen-II were measured with qRT-PCR. The levels of TNF-*α*, IL-6, IL-8, MMP-3, and MMP-13 were determined by ELISA. The protein levels of iNOs, COX-2, ADAMTS-4, ADAMTS-5, aggrecan, collagen-II, p-p65, p65, I*κ*B*α*, Nrf2, and HO-1 were assessed by Western blot.

**Results:**

Sappanone A inhibited the IL-1*β*-stimulated production of NO, PGE2, iNOS, COX-2, TNF-*α*, IL-6, and IL-8 in OA chondrocytes. In addition, sappanone A suppressed the expression of MMP-3, MMP-13, ADAMTS-4, and ADAMTS-5 in IL-1*β*-stimulated OA chondrocytes. The degradation of ECM components was reversed by sappanone A. Sappanone A prevented NF-*κ*B activation while enhanced Nrf2/HO-1 activation in IL-1*β*-treated chondrocytes.

**Conclusion:**

Sappanone A may be a potent therapeutic agent for OA.

## 1. Introduction

Osteoarthritis (OA) is a common progressive musculoskeletal disorder that mainly affects weight-bearing joints such as the knee and hip. The lesions include damage and loss of articular cartilage, reconstruction of subarticular bone, formation of bony redundancy, relaxation of the peripheral firmness band, and reduced muscle function [1]. The main symptoms of OA include pain, stiffness, and limited mobility of the joint. Pain in OA is usually classified as either persistent pain or intermittent severe pain that progresses over time. Osteoarthritis is currently one of the major disabling factors in the elderly and seriously affects the quality of life of patients [2]. According to statistics, there are approximately 300 million cases of osteoarthritis worldwide, and the prevalence continues to increase. As one of the most obvious risk factors for osteoarthritis, increasing age leads to a combination of individual exposure to risk factors and age-related biological changes in joint structure, resulting in an increased incidence of osteoarthritis. In addition to age, women, obesity, genetics, nutritional status, and history of trauma are also strong risk factors for osteoarthritis. Despite the more established risk factors associated with the risk of developing OA, little is known about the risk factors associated with the progression of OA, and the etiology of osteoarthritis is still unclear. Common treatment protocols include guidance for weight loss in overweight patients, nonsteroidal anti-inflammatory drugs for analgesia, and surgical treatment such as joint replacement [3].

RETRACTED

Previously, OA was considered a chronic overload and biomechanical impairment of the joint that impairs articular cartilage, resulting in stiffness, swelling, and loss of mobility. However, osteoarthritis was found to be a complex pathological process caused by inflammation and abnormal metabolism. During the course of osteoarthritis, the molecular composition of the articular cartilage matrix is altered, and the structural integrity of the tissue is disrupted. The lesion affects the deeper cartilage levels from the cartilage surface as the calcified cartilage area expands. As cartilage is repaired, hypertrophic chondrocytes exhibit a higher degree of activity. Throughout the pathological process, chondrocytes produce large amounts of matrix degradation products and proinflammatory mediators that act on the nearby synovial membrane to stimulate proliferation and inflammatory response. The proliferating synovial cells also release proinflammatory factors that exacerbate the response, while the subchondral bone shows an increased bone turnover rate and blood vessels cross the tidal line from the subchondral bone into the cartilage layer. Increased levels of inflammatory cytokines (mainly IL-1*β*) are found in synoviocytes and chondrocytes of OA patients [4]. It is known that IL-1*β* is one critical cytokine in OA progression [5], because it inhibits the production of extracellular matrix (ECM) components and induces the release of major extracellular proteolytic enzymes, such as MMPs and ADAMTSs, thereby promoting the cartilage degeneration [6].

Sappan Lignum is the dried material of Caesalpinia sappan L., family Leguminosae, with the efficacy of activating blood circulation and relieving swelling and pain. Modern pharmacological studies have shown that Sappan Lignum has anti-inflammatory, antibacterial, antitumor, antioxidant, hypoglycemic, and immunosuppressive activities. Sappanone A, one of the active ingredients of Sappan Lignum, can inhibit microglia activation in the brain and has a neuroinflammatory effect. Sappanone A is a homoisoflavanone with strong antioxidant and anti-inflammatory activities [7, 8]. Moreover, sappanone A pretreatment attenuates hypoxia-induced damage in PC-12 cells by inhibiting apoptosis [9]. A recent study showed that sappanone A protects myocardial cells from ischemia-reperfusion-caused injury through its anti-inflammatory effect via modulation of Nrf2 [10]. The study was performed to examine the biological influences of sappanone A on inflammation in OA chondrocytes when culture under IL-1*β* stimulation.

RETRACTED

## 2. Materials and Methods

### 2.1. Isolation and Intervention of Human OA Chondrocytes

Articular cartilage specimens from twelve OA patients (6 males, 6 females; aged 24-41 years) were obtained from The First Affiliated Hospital, College of Medicine, Xi'an Jiaotong University (Xi'an, CN). OA chondrocytes of cartilage samples were isolated as noted earlier [11]. The resulting cells were treated with incubation (37°C and 5% CO_2_) in 10% FBS-contained DMEM.

Human OA chondrocytes were adjusted to 1 × 10^5^ cells per well, followed by 2 h pretreatment with various concentrations of sappanone A. Subsequently, cells were given 24 h treatment (37°C) with IL-1*β* (10 ng/ml). Sappanone A (purity N98%) was purchased from ChemFaces (Wuhan, CN).

The study protocol and all amendments were approved by the appropriate ethics committee at each center. The study was done in accordance with the protocol, its amendments, and standards of Good Clinical Practice. All participants provided written informed consent before enrolment. Ethics number is MI-UI20200203.

### 2.2. Cell Viability Assay

Chondrocytes (5000 cells/well) were treated with 0, 5, 10, 20, or 40 *μ*M of sappanone A for 24 h. Then, the cells were incubated for 2 h with 10 *μ*l of CCK-8 solution, and the absorbance (450 nm) was detected.

### 2.3. qRT-PCR

Total RNA of chondrocytes obtained by TRIzol reagent (Invitrogen) was used for cDNA synthesis. The PCR reaction was carried out on CFX96 Real-Time PCR System (Bio-Rad). The mRNA levels of target genes were calculated using the 2^-*ΔΔ*Ct^ means, followed by normalization to GAPDH level.

### 2.4. Western Blot (WB)

Whole-cell lysates of chondrocytes were acquired for the following WB assay to determine the following proteins, including ADAMTS-4, iNOS, ADAMTS-5, COX-2, p-p65, aggrecan, p65, Nrf2, collagen-II, I*κ*B*α*, and HO-1. After separation by SDS-PAGE and transferring to Hybond-P membranes, the proteins were incubated with 1 : 500 diluted specific primary antibodies against the target protein (Thermo, USA) and 1 : 3000 diluted secondary antibody (Thermo). The signals were visualized using an enhanced chemiluminescence system (Thermo).

### 2.5. NO Assay

The Griess reaction approach was used to assess the NO concentration in culture medium using a commercial kit (Beyotime, CN). Samples were mixed with moderate Griess reagent, followed by a 10 min incubation without light. The absorbance (550 nm) was determined.

RETRACTED

### 2.6. ELISA

After treatment, culture supernatants of chondrocytes were acquired for the determination of IL-8, TNF-*α*, PGE2, IL-6, MMP-3, and MMP-13 concentrations using ELISA kits (R&D, USA).

### 2.7. Data Analyses

The normality of the sample was determined with the Shapiro–Wilk test. Descriptive statistical data were evaluated with the exploratory analyses of the Tukey test. Quantitative mean data (PES/WES, ISQ, and B.L.) were assessed with the nonparametric Wilcoxon-Mann–Whitney *U*-test to analyze the inferential statistical.

All data are presented by the mean ± SD. Significances among multiple groups were evaluated via the one-way ANOVA analysis of variance. *P* < 0.05 indicates a significant difference.

## 3. Results

### 3.1. Impact of Sappanone A on Cell Viability

The concentration of 40 *μ*M sappanone A produced a significant inhibitory effect on cell viability. Concentrations of 5, 10, and 20 *μ*M showed no significant change in cell viability. In the following experiments, the concentrations of 5, 10, and 20 *μ*M were used. (Figure 1).

### 3.2. Sappanone A Decreased NO and PGE2 Production

NO and PGE2 levels were significantly upregulated by 10 ng/ml IL-1*β* incubation. However, sappanone A significantly reduced the production of NO and PGE2 in IL-1*β* (10 ng/ml)-treated chondrocytes (Figure 2).

### 3.3. Sappanone A Repressed iNOS and COX-2 Expression

IL-1*β* stimulation led to the upregulated mRNA expression of COX-2 and iNOS. However, sappanone A decreased the mRNA expression of COX-2 and iNOS. Similarly, the protein expression of COX-2 and iNOS was increased with the stimulation by 10 ng/ml IL-1*β*; these effects were reversed by sappanone A pretreatment (Figure 3).

### 3.4. Sappanone A Inhibited Secretion of TNF-*α*, IL-8, and IL-6

The production of TNF-*α*, IL-8, and IL-6 was increased significantly in chondrocyte culture supernatants after intervention by 10 ng/ml of IL-1*β*, whereas sappanone A alleviated IL-1*β* caused increase in the production of TNF-*α*, IL-8, and IL-6 in a dose-dependent manner (Figure 4).

### 3.5. Sappanone A Attenuated the Expression of ADAMTSs and MMPs

Chondrocytes displayed significant upregulation in MMP-13 and MMP-3 production after intervention by 10 ng/ml IL-1*β*. However, sappanone A suppressed the MMP-3 and MMP-13 expression. IL-1*β* notably upregulated the protein levels of ADAMTS-5 and ADAMTS-4. Sappanone A remarkably inhibited the increase in protein levels (Figure 5).

### 3.6. Sappanone A Increased the Expression of Collagen-II and Aggrecan

The mRNA and protein levels of collagen-II and aggrecan were decreased significantly via IL-1*β* stimulation, while sappanone A markedly upregulated the levels of collagen-II and aggrecan in IL-1*β*-stimulated chondrocytes (Figure 6).

RETRACTED

### 3.7. Sappanone A Suppressed NF-*κ*B Activation

IL-1*β* notably increased the p-p65 level while decreased the I*κ*B*α* level. However, sappanone A presented a strong inhibition on IL-1*β*-induced changes in p-p65 and I*κ*B*α* expression levels. The results suggest that sappanone A inhibited IL-1*β*-treated NF-*κ*B signaling in chondrocytes (Figure 7).

### 3.8. Sappanone A Activated Nrf2/HO-1 Signaling

Sappanone A pretreatment promoted nuclear Nrf2 and HO-1 levels in chondrocytes in contrast to 10 ng/ml IL-1*β* treatment group (Figure 8). Thus, these data suggest that sappanone A took the anti-inflammatory effect through inducing the activation of Nrf2/HO-1.

## 4. Discussion

OA is a disease of the locomotor system caused by the degradation of the ECM, chondrocyte death, and bone redundancy, characterized by progressive damage to intra-articular cartilage, synovium, ligaments, and periarticular tissues. Current OA treatments are insufficient to arrest the progressive development of OA, and joint replacement is the only available alternative when progressing to advanced stages. Effective interventions for OA are instrumental in improving the quality of life of patients. OA is considered a mismatch disease caused by the body's inability to adapt to a new and rapidly changing environment and is a degeneration of joint tissue induced by a mismatch between genetics and the environment.

In addition to age-related effects, OA is also associated with a variety of factors such as exercise, obesity, metabolism, and diet, and the mechanisms of action and interrelationships of these relevant factors are poorly understood. The incidence of OA increases with age, and excessive mechanical stress loading of the joints due to excessive exercise and obesity and overweight may also contribute to the onset of OA. However, the association between aging and mechanical stress stimulation, two biological factors that persist in individuals, in the development of OA remains elusive. Inflammatory response with increased releasing of inflammatory cytokines participates in OA development [12, 13]. As a significant proinflammatory cytokine, IL-1*β* is involved in many inflammation-related diseases including OA. IL-1*β* action induces the production of different proinflammatory mediators from joint synovium and cartilage [14, 15]. In addition, IL-1*β* stimulation promotes the secretion of other proinflammatory cytokines, which may induce aggravated secondary insults [16]. The results of the present study found that sappanone A suppressed the production of TNF-*α*, PGE2, NO, IL-6, and IL-8 and downregulated iNOS and COX-2 expression. A previous study reported that sappanone A inhibited these inflammatory moleculars in RAW264.7 cells treated by LPS [17], which was consistent with the present study.

RETRACTED

OA is classified as “paralysis” in traditional Chinese medicine (TCM) and is caused by a deficiency of the liver and kidneys; cold and dampness invade the ligaments and remain in the joints, blocking the qi flow, resulting in dysregulation of the patient's qi flow, nondistribution of yang qi, numbness of the skin, and joint pain. Sappan Lignum has the effects of relaxing tendons, activating blood circulation, dispersing knots, sedating, dispelling blood stasis, and relieving pain. It is mainly used for fracture and tendon injury, bruises, stagnant swelling and pain, carbuncle and sores, heart and abdominal pain, blood stagnation and menorrhagia, postpartum stasis and abdominal pain, and dysmenorrhea. It also exhibits antitumor, antioxidant, anticomplement, anti-inflammatory, antibacterial, hypoglycemic, and immunosuppressive effects.

The release of ECM proteolytic enzymes is found to be increased under IL-1*β* stimulation [18]. MMPs, an important proteolytic system, are responsible for the degradation of ECM [19]. To the best of our knowledge, the inhibition of MMP production may prevent the cartilage degradation [20, 21]. ADAMTSs, expressed in mature articular cartilage, are also important proteolytic enzymes in OA [22]. Thus, medicines targeting MMPs and ADAMTSs may be viable OA therapies. Sappanone A significantly reduced the levels of MMPs and ADAMTSs in chondrocytes in our investigation. According to these findings, sappanone A possesses anti-inflammatory properties against OA. Many studies have shown that IL-1*β* stimulates the synthesis of ECM components by chondrocytes [23, 24]. Here, we found the capacity of sappanone A to prevent the degradation of aggrecan and collagen-II, which are major articular cartilage matrixes.

NF-*κ*B activation is a key process in OA through the regulation of proinflammatory moleculars [25]. I*κ*B-*α* masks the nuclear localization signals of NF-*κ*B proteins by maintaining them in cytoplasm at an inactive state, thereby inhibiting the NF-*κ*B activation [26]. Lee et al. [27] reported that sappanone A inhibited NF-*κ*B activation stimulated by LPS in RAW264.7 cells. Similarly, in the present study, sappanone A markedly suppressed NF-*κ*B activation in chondrocytes under IL-1*β* stimulation. Nrf2 is a critical transcription factor against oxidative damage [28]. Additionally, Nrf2 signaling also regulates the inflammatory response. Dysfunction of Nrf2 increases the risk of inflammatory diseases occurring [29–31]. The present study showed that sappanone A notably upregulated the protein levels of HO-1 and Nrf2 in chondrocytes.

RETRACTED

The study still has some limitations: the study only measured the indices at a single time point and did not consider the timeliness of sappanone A. The study design was flawed in that serum specimens were used for the detection of inflammatory factors, but not joint effusion or synovial tissue.

In conclusion, sappanone A suppressed the IL-1*β*-induced production of proinflammatory mediators and cytokines in OA chondrocytes. Sappanone A also suppressed the expression of ECM proteolytic enzymes and the degradation of ECM components. Mechanistic studies showed that sappanone A inhibited NF-*κ*B activation and induced Nrf2/HO-1 signaling.

## Figures and Tables

**Figure 1:** Cytotoxic effect of sappanone A on chondrocytes. The cytotoxicity of sappanone A on chondrocytes was detected by the CCK-8 assay. ^∗^*P* < 0.05 compared to control group.

**Figure 2:** Sappanone A decreased IL-1*β*-induced production of NO and PGE2 in chondrocytes. (a) Griess method for NO concentration analysis. (b) ELISA for PGE2 concentration analysis. ^#^*P* < 0.05 compared to control group and ^∗^*P* < 0.05 compared to IL-1*β* treatment group.

**Figure 3:** Sappanone A suppressed IL-1*β*-induced expression of iNOS and COX-2 in chondrocytes. (a, b) qRT-PCR analysis for the iNOS and COX-2 mRNA expression. (c, d) WBting analysis for the iNOS and COX-2 protein expression. ^#^*P* < 0.05 compared to control group and ^∗^*P* < 0.05 compared to IL-1*β* treatment group.

**Figure 4:** Sappanone A inhibited IL-1*β*-induced production of TNF-*α*, IL-6, and IL-8 in chondrocytes. (a) TNF-*α*, (b) IL-6, and (c) IL-8 concentration was determined by ELISA. ^#^*P* < 0.05 compared to control group and ^∗^*P* < 0.05 compared to IL-1*β* treatment group.

**Figure 5:** Sappanone A attenuated the expression of MMPs and ADAMTSs in IL-1*β*-induced chondrocytes. (a) MMP-3 and (b) MMP-13 concentration was determined by ELISA. The protein expression levels of (c) ADAMTS-4 and (d) ADAMTS-5 were assessed by WB. ^#^*P* < 0.05 compared to control group and ^∗^*P* < 0.05 compared to IL-1*β* treatment group.

**Figure 6:** Sappanone A increased the levels of aggrecan and collagen-II in IL-1*β*-induced chondrocytes. (a, b) qRT-PCR analysis for the aggrecan and collagen-II mRNA expression. (c, d) WBting analysis for the aggrecan and collagen-II protein expression. ^#^*P* < 0.05 compared to control group and ^∗^*P* < 0.05 compared to IL-1*β* treatment group.

RETRACTED

**Figure 7:** Sappanone A suppressed IL-1*β*-induced NF-*κ*B activation in chondrocytes. WBting analysis for the protein levels of p-p65, p65, and I*κ*B*α*. ^#^*P* < 0.05 compared to control group and ^∗^*P* < 0.05 compared to IL-1*β* treatment group.

**Figure 8:** Sappanone A activated Nrf2/HO-1 signaling pathway in IL-1*β*-induced chondrocytes. Western blotting analysis for the protein levels of Nrf2 and HO-1. ^#^*P* < 0.05 compared to control group and ^∗^*P* < 0.05 compared to IL-1*β* treatment group.

## Data Availability

All data generated or analyzed during this study are included in this published article.
